The article "Fluid-Solid Coupling Simulation of Wall Fluid Shear Stress on Cells under Gradient Fluid Flow" was published in 2021. Journal: Appl Bionics Biomech.

# Fluid-Solid Coupling Simulation of Wall Fluid Shear Stress on Cells under Gradient Fluid Flow

**DOI:** 10.1155/2021/8340201

**Published:** 2021-12-02

**Authors:** Xiao Zhang, Yan Gao, Bo Huo

**Affiliations:** Biomechanics Lab, Department of Mechanics, School of Aerospace Engineering, Beijing Institute of Technology, Beijing 100081, China

## Abstract

Fluid shear stress (FSS) plays a crucial role for cell migration within bone cavities filled with interstitial fluid. Whether the local wall FSS distribution on cell surface depends on the global gradient FSS of flow field should be clarified to explain our previous experimental observation. In this study, finite element models of discretely distributed or hexagonal closely packed cells adherent on the bottom plate in a modified plate flow chamber with different global FSS gradient were constructed. Fluid-solid coupling simulation of wall fluid shear stress on cells was performed, and two types of data analysis methods were used. The results showed that the profile of local FSS distribution on cell surface coincides with the angle of cell migration determined in the previous study, suggesting that RAW264.7 osteoclast precursors may sense the global FSS gradient and migrate toward the low-FSS region under a high gradient. For hexagonal closely packed cells, this profile on the surface of central cells decreased along with the increase of cell spacing, which may be caused by the higher local FSS difference along the direction of FSS gradient in the regions close to the bottom plate. This study may explain the phenomenon of the targeted migration of osteoclast precursors under gradient FSS field and further provide insights into the mechanism of mechanical stimulation-induced bone remodeling.

## 1. Introduction

Bone remodeling is an important physiological process characterized by bone formation and bone resorption [1, 2]. The structure of bone tissue under mechanical loading could be optimized through the process called as bone remodeling to adapt to the change in mechanical environment [3]. Many studies showed that under mechanical loading, the fluid flows within bone cavities, such as Harversian canals or the lacunar-canalicular system, and the corresponding fluid shear stress (FSS) is the main factor for producing biological response in bone cells [4, 5]. As in vivo fluid in bone cavities is difficult to directly observe, some in vitro loading devices were constructed to exert fluid flow on cells. Compared with cone-and-plate flow chamber [6–8], parallel-plate flow chamber is widely used to produce wall FSS in vitro on cells due to its advantage of controlling the FSS field [9–11].

In the previous study of the authors, a modified plate flow chamber, in which the top cover is not parallel to the bottom plate in the direction perpendicular to the longitudinal axis of the chamber, was constructed [12]. Finite element analysis (FEA) showed that this device was able to provide a global FSS field with gradient on the bottom plate [13]. The striking experimental results demonstrated that osteoclast precursors RAW264.7 under globally gradient FSS migrated towards the region with low wall FSS rather than along the flow direction. This seems to be a unique ability for osteoclasts because other four types of cells, i.e., osteoblast-like MC3T3-E1 cells, periodontal ligament fibroblasts, rat mesenchymal stem cells, and Madin-Darby canine kidney epithelial cells, migrate along flow direction but not responding to FSS gradient [6]. However, the mechanism of this FSS gradient-dependent migration is still unknown.

The article "Fluid-Solid Coupling Simulation of Wall Fluid Shear Stress on Cells under Gradient Fluid Flow" was published in 2021. Journal: Appl Bionics Biomech.

Some studies demonstrated that the intracellular calcium signaling pathways may influence the migration of osteoclast precursors under fluid flow [6, 12, 14–16]. One previous study has found that the directional movement of a cell may be influenced by the front-to-rear polarization of intracellular calcium [17]. Therefore, we speculated that this global fluid field with FSS gradient around cells leads to similar gradient distribution of local FSS on cell surface, then triggers mechanosensitive cation channel (MSCC) in the cell membrane by different levels of membrane tension caused by local FSS at different locations on cell surface; further, there may be different amount of extracellular calcium ions entering cytoplasm through MSCC at different location, and the gradient of intracellular calcium concentration may result in the migration of osteoclasts toward low FSS region. Therefore, a reasonable hypothesis is that the polarization of wall FSS on a cell may correlate with that of membrane tension and intracellular calcium concentration, which finally determines the extent of cell migration opposite to the FSS polarization direction.

In the present study, the FSS distribution on cell surface is mainly assumed to characterize directional migration via a series of Ca^2+^ signaling pathways. Finite element (FE) models with discretely distributed or hexagonal closely packed cells on the bottom plate of modified plate chamber were first constructed. Then, the effect of different FSS magnitudes and gradients as well as cell spacing on the local distribution of wall FSS on cell surface was investigated. Finally, the polarization level of wall FSS on a cell was compared with the level of cell migration found in the previous study.

## 2. Materials and Methods

### 2.1. FE Model of Modified Plate Chamber

A modified plate flow chamber was developed in the lab to provide flow field with different gradients of wall FSS on the bottom plate (Figure 1(a)). The difference of this device compared with a traditional parallel-plate flow chamber is the leaning top cover that is not parallel to the bottom plate along the direction perpendicular to the longitudinal axis of the chamber [12] (Figures 1(b) and 1(c)). The dimensions of flow channel are 12 mm in width (*w*), 50 mm in length (*l*), and 0.2 mm in height (*h*1) at one side, and 0.8 mm in height (*h*2) at the other side. The wall FSS on the cell surface could be controlled by specifying the rotation speed of a peristaltic pump. Then, hexagonal closely packed single cell or group cells with 10 *μ*m in radius, which is nearly actual size of RAW264.7 osteoclast precursor, were placed at different positions on the bottom plate (Figures 1(d)–1(f)); these cells are in the same location as those observed in the previous experimental study [12].

The article "Fluid-Solid Coupling Simulation of Wall Fluid Shear Stress on Cells under Gradient Fluid Flow" was published in 2021. Journal: Appl Bionics Biomech.

### 2.2. Material Property of Cells

In this study, the hyperelastic model with compressible isotropic Hookean material property was adopted for the cells. A simple nonnegative strain energy density for a compressible isotropic Hookean material was proposed as follows [18]:

(1) $$\begin{array}{c} W_{s}=\frac{1}{2}G\left(I_{\lambda }-3\right)+\frac{1}{2}\Lambda {\left(\ln J\right)}^{2}-G\ln JdV, \end{array}$$

where the material constants are defined by

(2) $$\begin{array}{c} G=\frac{E}{2\left(1+\mu \right)},\text{and }\Lambda =\frac{E\mu }{\left(1+\mu \right)\left(1-2\mu \right)}. \end{array}$$

In the above expression, *E*, *G*, *μ*, and *Λ* denote the elastic modulus, shear modulus, Poisson's ratio, and the Lamé constant, respectively. The Poisson's ratio must be less than 0.5 and greater than −1 to guarantee that the strain energy density is positive for all deformations.  Table 1 presents the specific material properties for the cells used in this study.

### 2.3. Computational Fluid Dynamic Simulation

Steady fluid flow simulation based on FEA was performed on the modified flow chamber by using COMSOL Multiphysics software. Fluid flow was simulated with laminar flow of low Reynolds number, and no-slip boundary condition was assumed for all rigid surfaces in the model. The fluid was assumed to be viscous and incompressible with density (*ρ*) of 1 × 10^3^ kg/m^3^ and viscosity of 1 × 10^−3^ Pa × s. The inlet pressure was assigned as 300 Pa and the outlet pressure as 0, 100, and 200 Pa, corresponding to three FSS gradients of 0.2, 0.10, and 0.05 Pa/mm, respectively. The above pressure differences are similar to those in lacunar-canalicular system with the bone [21]. For a steady flow and the hyperelastic model of cells, the equations were solved using an iterative method, and the convergence was identified when the relative tolerance was less than 0.001.

The article "Fluid-Solid Coupling Simulation of Wall Fluid Shear Stress on Cells under Gradient Fluid Flow" was published in 2021. Journal: Appl Bionics Biomech.

### 2.4. Data Analysis

The dorsal surface of each cell was divided into four sectors, including the sector with the higher global FSS (SHFSS) and the opposite one with the lower global FSS (SLFSS), to reveal the distribution of local wall FSS on cell surface relative to the direction of the global FSS gradient (as shown in Figure 2(f)). In addition, two types of data analysis methods, i.e., calculating the average FSS values in whole SHFSS and SLFSS regions and in the bands with orientations of 30°, 45°, and 60° relative to the sphere center, were established (Figures 2(g) and 2(h)). The ratios of the average value (RAV) of local FSS in SHFSS relative to that in SLFSS at seven *y* locations with the same *x* location were calculated. The positive RAV indicates that more MSCC in SHFSS region may be activated than those in SLFSS region, which may further lead to polarized distribution of intracellular calcium ions and the low-FSS migration. In contrast, the RAV close to zero reveals that the cells tend to migrate along flow direction. MATLAB and Origin software were used for data processing.

## 3. Results and Discussion

### 3.1. Novel Plate Flow Chamber Provides Flow Field with Gradient FSS

The mesh sensitivity test revealed that when the number of total elements was bigger than 175,000, the wall FSS on the cell surface converged (Figure 2(a)). The FEA results based on this model obviously showed a FSS gradient along the direction perpendicular to the flow direction. When the pressure difference at the inlet and outlet of flow chamber was changed, three FSS gradients, 0.05, 0.1, and 0.2 Pa/mm, were produced (Figures 2(b) and 2(c)). Statistical analysis further verified that the wall FSS has a linear relationship with the distance along the FSS gradient (Figure 2(d)). The velocity at the same height along the flow direction showed that it is nearly constant at the same height (Figure 2(e)). The above result indicated that a flow field with gradient FSS was constructed.

### 3.2. RAV Is Dependent on FSS Magnitude and Gradient for Discretely Distributed Cells

The FSS around the cells numerically simulated with the same location as those in the previous experiment for the cells to experience FSS with same magnitude and gradient [12]. Furthermore, seven positions along *y* direction from 10 mm to 40 mm with intervals of 5 mm were chosen for placing the cells in the FE model (Figure 3(a)). When each cell was placed at these specified positions, the FSS on the top region of the cells was obviously higher than that close to the adhesion region (Figures 3(b) and 3(c)). Then, we compared the effect of different FSS magnitude on RAV of each cell under different FSS gradient. In the 0.05 Pa/mm group, the RAV was independent of FSS magnitudes of 0.1, 0.4, and 0.8 Pa (Figure 3(d)). However, in the 0.1 and 0.2 Pa/mm groups, the RAV significantly decreased with the increase in FSS magnitude (Figures 3(e) and 3(f)). The relation between the RAV of cells and the FSS gradient was further studied for the two FSS levels of 0.1 Pa and 0.8 Pa, which are in the physiological range of FSS in the postcapillary venules or osseous lacunae [12]. For 0.1 Pa FSS, the RAV under 0.2 Pa/mm was significantly greater than that under 0.05 and 0.1 Pa/mm. However, the RAV under 0.1 and 0.2 Pa/mm decreased compared with that under 0.05 Pa/mm (Figures 3(d)–3(f)). Therefore, the above results showed that the migration of cells toward the low-FSS region in a flow field with gradient FSS, especially when the FSS magnitude is relatively low.

The article "Fluid-Solid Coupling Simulation of Wall Fluid Shear Stress on Cells under Gradient Fluid Flow" was published in 2021. Journal: Appl Bionics Biomech.

### 3.3. RAV on Central Cells Is Dependent on FSS Magnitude and FSS Gradient for Hexagonal Closely Packed Cells

In order to describe the effect of different cell spacing on a cell in the case of multiple cells, the hexagonal closely packed arrangement with three different cell spacings, i.e., 2 *μ*m (representing the cells approaching each other), 20 *μ*m (one cell spacing), and 40 *μ*m (two cell spacing), were constructed in different locations along the flow direction to study the effect of neighbouring cells on the local FSS field on the cell surface (Figure 4(a)), and only the central cells were analyzed. The results showed that under the same FSS gradient, the RAV of the cells at the location of low FSS amplitude decreased first and then increased along with cell spacing, thus forming a U-shape distribution (Figures 4(h)–4(j)). This trend became more pronounced with the increase in FSS gradient. When the FSS magnitude gradually increased, this tendency gradually changed as a linearly decreasing distribution (Figures 4(c) and 4(d)). Decreasing cell spacing may enhance the polarization distribution of the wall FSS on the cell surface more than the discrete cells.

### 3.4. RAV Close to Adhesion Region Is Higher than the Top Region

Three bands on the cell surface with different orientations were considered, i.e., 30°, 45°, and 60°, to explain which part in SHFSS and SLFSS dominates the RAV difference for the cells (Figure 5(a)). Under three FSS gradients, the RAV of the central cell at 30° band was significantly greater than that at 45° and 60° bands. As the FSS gradient and cell spacing increased, the local FSS revealed a linearly decreasing distribution (Figures 5(b)–5(m)). In addition, when the cell spacing was small, the RAV of the central cell at 30° band was larger than that with bigger cell spacing, including the case of discrete distribution. Therefore, the RAV of the central cell at 30° band may play a key role in regulating cell migration against the direction of FSS gradient.

The article "Fluid-Solid Coupling Simulation of Wall Fluid Shear Stress on Cells under Gradient Fluid Flow" was published in 2021. Journal: Appl Bionics Biomech.

## 4. Conclusions

This study is aimed at explaining the previous experimental observation that osteoclast precursors move towards the low-FSS area in the gradient FSS field, evidently deviating from the direction of fluid flow5. The modified plate flow chamber was mimicked using FEA to construct the gradient FSS field, and hyperelastic cells were discretely distributed or hexagonal closely packed on the bottom plate with gradient FSS. The polarization distribution of the local wall FSS on the cell surface was compared with the experimental results of cell migration.

Several arrangements of cells on the plate were investigated in this study. First, discretely distributed cells were arranged along the flow direction and exposed to a gradient FSS field with the FSS magnitude ranging from 0.1 Pa to 2.0 Pa, which was the physiological level within the bone cavities [7]. The discrete distribution of cells was to mimic the case that no intercellular interaction was present on the wall FSS on the cell surface. For the FSS gradient of 0.05 Pa/mm, the RAV of each cell was independent of FSS magnitude. When the FSS gradient was increased up to 0.1 and 0.2 Pa/mm, the RAV decreased approximately linearly with the FSS magnitude increased. In particular, for the constant FSS magnitude of 0.1 Pa, the RAV obviously increased along with FSS gradient. Interestingly, the relation of RAV of the local wall FSS on cells with FSS magnitude and gradient is similar to the experimental results of migration angle of RAW264.7 cells, i.e., migrating opposite to the direction of FSS gradient towards the low-FSS region in a flow field with gradient FSS especially when the FSS magnitude was relatively low and the FSS gradient was relatively high [12]. Therefore, the local wall FSS may be the main driving factor of targeted migration of osteoclast precursors under gradient FSS flow field.

For hexagonal closely packed assignment with different cell spacings under three different FSS gradients, at low FSS magnitude, the RAV showed a U-shape curve along with the increase in cell spacing, which is independent of FSS gradient. For high FSS magnitude, this U-shape profile shifted, and the relation between RAV and cell spacing tended to be linear, i.e., RAV decreased when cells were gradually away from one another. Three bands with different orientations were considered to further clarify which part of the cell surface regulates RAV under gradient FSS. The results indicated that the RAV at the 30° band of central cells was significantly greater than that at 45° and 60° bands, suggesting that the RAV close to the adhesion region on the cell surface played a key role to regulate the migration of RAW264.7 cells opposite to the direction of FSS gradient.

The article "Fluid-Solid Coupling Simulation of Wall Fluid Shear Stress on Cells under Gradient Fluid Flow" was published in 2021. Journal: Appl Bionics Biomech.

In summary, the FEA results in this study showed that the gradient FSS field led to the polarization distribution of local FSS on the cell surface, and decreased cell spacing increased this phenomenon. The above phenomenon was dependent on FSS's magnitude and gradient. The difference in local FSS on the cell surface under the gradient FSS field may be the fundamental reason for the migration of osteoclast precursors towards the low-FSS region.

## Figures and Tables

**Figure 1:** Establishment of gradient parallel plate flow chamber and FE model. (a) Photo of custom-made gradient flow chamber, in which the arrow represents the direction of FSS gradient. Schematics of gradient flow chamber in cross-sectional view (b) and side view (c). (d) FE mesh indicated by the blue box in (a). (e) FE mesh around a cell indicated by the green box in (d). (f) FE mesh of the cell indicated by the yellow box in (e).

**Figure 2:** Analytical method of wall FSS on cell surface. (a) Mesh dependency analysis. (b) FE mesh and wall FSS of gradient flow chamber. (c) Numerical simulation results of wall FSS on the bottom plate at the location indicated by the red box in (b). (d) Wall FSS of all nodes at different FSS gradients and linearly fitted by the dotted line. (e) Fluid velocity of the locations with the same height of 0.4 mm and two different x positions. (f) Dorsal surface of a cell divided into four sectors, including the sectors with higher global FSS (SHFSS) and lower global FSS (SLFSS). (g) Bands on the cell surface with three orientations, i.e., 30°, 45°, and 60°. (h) Top views of the bands with different orientations in the sectors.

**Figure 3:** Average wall FSS in SHFSS and SLFSS on discretely distributed cells along flow direction. (a) Schematic of the cells arranged on the bottom plate with different locations. (b) Top and (c) side views of wall FSS on cell surface. (d–f) Ratios of average value (RAV) of local FSS in SHFSS relative to that in SLFSS; ^∗^*p* < 0.05.

**Figure 4:** RAV on hexagonal closely packed cells. (a) Schematic of hexagonal closely packed cells with different cell spacings. (b, e, and h) RAV on central cell at three FSS magnitudes under constant FSS gradient of 0.05 Pa/mm. (c, f, and i) RAV on central cell at three FSS magnitudes under constant FSS gradient of 0.1 Pa/mm. (d, g, and j) RAV on central cell at three FSS magnitudes under constant FSS gradient of 0.2 Pa/mm.

The article "Fluid-Solid Coupling Simulation of Wall Fluid Shear Stress on Cells under Gradient Fluid Flow" was published in 2021. Journal: Appl Bionics Biomech.

**Figure 5:** RAV within the bands of different orientations on hexagonal closely packed cells. (a) Schematic of hexagonal closely packed cells. (b, e, h, and k) RAV within the bands with different orientations on central cell at three FSS magnitudes under constant FSS gradient of 0.05 Pa/mm. (c, f, i, and l) RAV within the bands with different orientations on central cell at three FSS magnitudes under constant FSS gradient of 0.1 Pa/mm. (d, g, j, and m) RAV within the bands with different orientations on central cell at three FSS magnitudes under constant FSS gradient of 0.2 Pa/mm.

**Table 1:** Parameters used in the FEA.

Material property	Values for osteoclast precursors
Density of a cell (*ρ*, kg/m^3^)	1100 [19]
Poisson's ratio (*μ*)	0.3 [4]
Young's modulus (*E*, N/m^2^)	5000 [20]
Lamé constant (*Λ*, N/m2)	2885
Shear modulus (*G*, N/m2)	1923

## Data Availability

The data used to support the findings of this study are available from the corresponding author upon request.
